# An ANP‐fuzzy evaluation model of food quality safety supervision based on China's data

**DOI:** 10.1002/fsn3.1561

**Published:** 2020-06-05

**Authors:** Xiuhua Zhang, Jun Zhang, Tingqiang Chen

**Affiliations:** ^1^ School of Foreign Language Zhengzhou University of Aeronautics Zhengzhou China; ^2^ School of Economics and Management Nanjing Tech University Nanjing China

**Keywords:** analytic network process, empirical research, food safety, fuzzy comprehensive evaluation method, supervision performance

## Abstract

A government acts as the main supervisor of food quality and safety. How to quantify and improve the performance and efficiency of government supervision, respectively, is an urgent problem. This study constructs a food safety supervision performance index and utilizes an analytic network process‐fuzzy comprehensive evaluation model to precisely quantify the performance of government supervision. The evaluation results show that, (a) although the overall situation of food quality and safety in China is controllable, the government does not do well in food safety risk supervision, food recall supervision, and accident summary supervision. (b) Internal supervision is the weakest link in food quality and safety supervision. (c) Grassroots supervision is weak especially in prefecture and county levels. (d) There is no positive correlation between the economy level and supervision level in one region. This paper contributes to accurately reflecting the status quo of China's food safety supervision and realizing the transparency of government regulatory information, which ultimately boosts the government's efficiency in food safety supervision and improves the regulatory situation.

## 1 INTRODUCTION

Improving the efficiency of government supervision and strengthening supervision has become a hot topic in the field of food safety supervision since the outbreak of the "poisonous milk powder" incident in 2008. On the one hand, the quality of public life is improving, and the supply‐side enterprises urgently need to improve food quality(Cao, Tian, & Wang, 2013; Jongwanich, 2009; Liu & Niyongira, 2017), On the other hand, although the current situation of food safety in China is generally stable^0^, there are still a lot of problems. Constantly exposed food safety incidents, from “Fuxi overdue meat” event in 2014, “fake milk powder “incident in 2016 until “nuclear pollution food” events in 2017, stimulate the nerve of the public0. At the same time, they also arouse public suspicion of government efforts on food safety supervision and test government capacity and credibility0.

In China, the frequent food safety accidents not only had technical reasons, but also deep‐seated management issues0, which included information asymmetry in the food market, the imbalance interests between various stakeholders in the industry chain during evolution game and the lack of supervision0. Market failure caused by information misalignment was an important reason for food safety problems, manufacturers could use this asymmetry and take opportunistic behavior, which caused serious moral hazard0. On the supply side, manufacturers could cause food safety risks spread rapidly along the food supply chain to the downstream, leading to food safety incidents (Chen, Ma, & Wang, 2018; Wang & Chen, 2016). In addition, current society cogovernance system for food safety in China has not yet been established (Zhang & Xue, 2016; Zhou, Yang, & Wu, 2016), and the regulatory role of the public forces such as consumers and the media cannot be fully implemented, so as to failures to prohibit food safety problems repeatedly.

According to the definition of the international organization, food safety regulation, also known as food control, refers to the mandatory legal action carried out by the government departments in order to protect the legal rights of the consumers, ensure that food is consistent with food safety and quality requirements from production to sale (FAO & WHO, 2003). The government, as the core department, has the main responsibility for the supervision of safe food. However, there are still some problems in the practice of food safety supervision in China. Initially, the law system of food safety in China is not perfect0). With the development of society, the emerging food safety issues are not covered by food safety regulations, which brings difficulties to the government supervision and law enforcement, leading to the poor supervision effect. Furthermore, food recall machine and risk monitoring and assessment of food safety in China is still in the exploration stage (Michaud et al., 2001; Xia & Tonsor, 2017), resulting in consumers having difficulty obtaining information related to food safety. Additionally, the scientific performance appraisal mechanism of government departments has not been established (Zhou et al., 2016). Far from seriously performing their duties of protecting the safety of consumer, law enforcement authorities will be "captured" by food enterprises (Jia & Jukes, 2013; Laffont & Tirole, 1990; Lam, Remais, & Fung, 2013), causing the failure of administrative supervision.

At present, research on government performance is scant, and very few scholars adopted the quantitative analysis method to evaluate the government's food safety supervision performance (FSSP) level. The network process‐fuzzy comprehensive evaluation model is a good method to evaluate the government's food safety supervision performance (FSSP) level. On the one hand, the evaluation indicators of the government's food safety regulatory performance are complex, multi‐attribute and interrelated, and ANP can be used to systematically evaluate such a relevant multi‐indicator system (Pang & Bai, 2013). On the other hand, the evaluation of the government's food safety regulatory performance is difficult to be quantified with precise figures, and the fuzzy comprehensive evaluation model can be used to study this ambiguous situation (Annadurai, Babu, & Srinivasamoorthy, 2000). Consequently, from the perspective of multi‐link supervision, based on the analysis of food safety regulations and existing literatures, this study constructs the food safety evaluation index system through the network process‐fuzzy comprehensive evaluation model. A total of 690 questionnaires containing 20,010 data are collected from food and drug administration (FDA hereinafter). In China, FDA is the official government department that is in charge of food and drug management and supervises the implementation of various systems and standards under the subordinate local governments according to the laws and regulations at the central, provincial, prefectural, and county levels. Basing on these data, the FSSP level is evaluated.

The rest of the paper is organized as follows. Section 2 presents the setup of the index system of FSSP. Section 3 introduces the fuzzy‐ANP comprehensive evaluation model and analyzes its applicability. Section 4 discusses an empirical research and analyzes the results of the empirical study. Finally, Section 5 includes research findings, deficiencies, and future research directions.

## 2 CONSTRUCTION OF EVALUATION INDEX

Food safety supervision is a systematic engineering which involves presupervision, internal supervision, and postsupervision (Ma, 2015). Frequent food safety accidents expose the government's deficiencies in food safety supervision (Li, 2011). For that reason, the state has formulated a number of relevant laws and regulations. Meanwhile, evaluating the performance of local governments’ food safety supervision is becoming an important means for the central government, which urges the local governments to implement the relevant laws and regulations on food safety (Liu & Niyongira, 2017). Thus, the following three aspects can be considered in improving FSSP.

### 2.1 Presupervision

Presupervision refers to regular supervision measures and food safety risk warning mechanisms made by government, so as to prevent the occurrence of food safety incidents. Therefore, it can be divided into the following two aspects:

#### 2.1.1 Regular supervision of food safety

Regular supervision of food safety focuses on effective actions to solve routine problems (Chen, 2011). According to the existing achievements and the Food Safety Law of the People's Republic of China (2015 Revision) (FSL hereinafter), to evaluate FSSP, the regular supervision of food safety can be subdivided into three indexes, namely, publicity of public welfare of food safety, compulsory insurance coverage of food safety liability, and declaration of the state of national food safety standards0; (Chen, 2011; Pei et al., 2011; Qi, 2013; Trienekens & Zuurbier, 2008).

#### 2.1.2 Food safety risk supervision

Establishing and improving the food safety risk prevention system are conducive to alleviate the food safety risk of market failure and achieve the social optimum of food safety. According to the existing achievements and the FSL, food safety risk supervision can be divided into four indexes to evaluate FSSP, which include established situations of a risk monitoring system for food safety, of a risk assessment system for food safety, and of a risk communication system for food safety and coverage situations and to check the frequency of food varieties yearly0.

### 2.2 Internal supervision

Internal supervision is the food recall supervision and accident control regulation carried out during the food safety accident, so as to prevent the diffusion of food safety hazards and reduce the negative impacts of it. It focuses on the implementation of various regulatory policies and legal systems (Wang & Chen, 2016). Therefore, it can be divided into the following two aspects.

#### 2.2.1 Food recall supervision

Improving the food recall system is helpful in changing the situation of China's food safety0. With the food recall system, the government will minimize food safety hazards by taking coercive measures or guiding enterprises to recall defective food that threaten consumers’ health (Han, 2014). According to the existing results and the FSL, food recall supervision can be subdivided into six indexes to evaluate FSSP, namely, establish situation of a food recall system, timeliness of food recall, availability of food recall explanation, food recall explanation comprehensibility, recording the name and specification of unsafe food, and remedial or destructed situation of recalled unsafe food 0).

#### 2.2.2 Food safety accident control supervision

In view of the outbreak of food safety accidents, the government must immediately set up a food safety accident handling command organization and start contingency plans (Li, 2011; Lin, 2009) and do a good job of organization and coordination, information communication and other aspects of the work. According to the existing results and the FSL, food safety accident control supervision can be subdivided into five indexes to evaluate FSSP, namely, establish situation of commanding food safety accident management headquarters, professionality of emergency disposal personnel of food safety accidents, handling of food safety accident work timeliness, timeliness of published warning information of food safety, and accuracy of the published warning information of food safety (Gong, Zhang, & Yu, 2013; Li, 2011; Lin, 2009; Pan & Xu, 2013).

### 2.3 Postsupervision

As the last link of the entire supervision process, postsupervision is mainly the summary and investigation of the cause of accidents and the attribution of responsibilities. It aims to promoting the perfection of the food safety regulation system (Henderson, Coveney, & Ward, 2010). Therefore, it can be divided into the following two aspects.

#### 2.3.1 Food safety accident summary supervision

The government should carry out a summary of accidents, to optimize the regulation system (Li, 2011; Lin, 2009) and enhance its capacity to prevent and respond to similar food safety accidents in the future. According to the existing results and the FSL, food safety accident summary supervision can be subdivided into seven indexes to evaluate FSSP, namely, conducting an epidemiological investigation of factors related to the food safety incident, declaring investigation on an incident and handling information of food safety accidents, recording the situation in food safety credit records, adjusting to the frequency of supervision and inspection of food producers and distributors, talking with legal representatives whose company has hidden dangers, investigating the situation for traceability of the accidents, and optimizing the situation of the postsupervision system (Li, Liu, & Sun, 2015; Sun & Wang, 2015; Zhou & Wang, 2012).

#### 2.3.2 Food safety accident investigation supervision

Many food safety accidents in China are directly related to the dereliction of regulatory bodies (Zhu & Xie, 2014). Improving the investigation of major liability accidents is helpful to conduct a fair, responsible and comprehensive investigation and punish those who are deaf to the laws in the field of food safety (Sui, 2009). According to the existing achievements and the FSL, the food safety accident investigation supervision can be subdivided into four indexes to evaluate FSSP, which include investigation of the liabilities of the organization where the food safety accidents occurred, investigation and certification of the people from regulatory authorities who are involved in dereliction of their duty, and impartiality and comprehensiveness in the investigation of the responsible parties of these food safety accidents (Connolly, Luo, Woolsey, Lyons, & Phillips‐Connolly, 2015; Du, 2012; Sui, 2009; Zhu & Xie, 2014).

In light of the all above considerations, by combining the opinions from Delphi expert group which consists of food safety management professors from different colleges and universities and experts in FDA, food business and food safety media, this study systematically reviews the classic literature of FSSP evaluation and the latest laws and regulations, and establishes the index system of FSSP, as shown in Table S1 refer to appendix.

## 3 EVALUATION MODEL

The ANP‐fuzzy comprehensive evaluation model is composed of analytic network process (ANP) (Saaty, 2012) and fuzzy comprehensive evaluation method. On the one hand, compared with analytic hierarchy process (AHP), ANP can effectively measure the interaction between different decision‐making layers or different indexes in the same layer. On the other hand, based on the membership degree theory in fuzzy mathematics, the fuzzy comprehensive evaluation method can effectively achieve a quantitative evaluation of qualitative indexes.

This paper utilizes the ANP‐fuzzy comprehensive evaluation model to evaluate the FSSP mainly based on the two following considerations: (a) There exists an obvious hierarchical structure between the same supervision links and a strong interdependence between different regulatory links in the index system of FSSP. (bb) Individual indexes are difficult to quantify, and the values are characterized by interval and ambiguity in the index system of FSSP. Thus, using the ANP‐fuzzy comprehensive evaluation model to evaluate the FSSP is scientific and practical. Accordingly, this method is widely applied to transportation and international investment (Huang, 2012; Onut, Tuzkaya, & Torun, 2011).

### 3.1 Constructing the network structure of ANP

The network structure of FSSP consists of the control and network layers. The control layer contains the target and criteria: The target is A (FSSP), and the criteria are the first‐level indexes of the index system namely B_1_, B_2_, and B_3_. The network layer consists of six sets of elements that correspond to the second‐level indexes, and the third‐level indexes in the index system, specifically C_1_, C_2_, C_3_, C_4_, C_5_, and C_6_. According to the interdependence relationship among the elements of the index, the network structure of ANP is constructed (Figure 1).

**Figure 1:** Network structure of ANP of FSSP

### 3.2 Determination of the index weight

Based on ANP and Delphi expert scoring, the weight of each FSSP indexes is obtained. The detailed steps are as follows:

Step 1: calculate a super matrix and weighted super matrix. Suppose that ANP control layer criterion contains first‐level index $P_{S}\left(s=1,2,\cdots ,m\right)$, the network layer contains second‐level index $C_{S}\left(s=1,2,\cdots ,n\right)$. According to the criterion of the control layer element $P_{S}$, determine the interaction between the secondary indexes. Then, construct the judgment matrix and obtain the normalized feature vector ${\left(w_{i1},w_{i2},\cdot \cdot \cdot ,w_{\mathrm{im}}\right)}^{T}$. Furthermore, test the consistency of the obtained vector and get a super matrix $W_{\mathrm{ij}}$.Thus, the super matrix W can be obtained under the criterion $P_{S}$, as is shown in formula (1). Finally, normalize the column vector of super matrix and get a weighted super matrix $\bar{W}$.

(1) $$W=\left[\begin{array}{cccc} W11 & W12 & \cdots & W1n\\ W21 & W22 & \cdots & W2n\\ \vdots & \vdots & \vdots & \vdots \\ Wm1 & Wm2 & \cdots & \mathrm{Wmn} \end{array}\right]$$

Step 2: The ANP limit matrix $W^{\infty }$, as is shown in formula (2), is obtained by stabilizing the weighted super matrices. If the limit is convergent and unique, the column vector in the matrix is the stable weight of each FSSP indexes.

(2) $$W^{\infty }=\lim_{i\to \infty }\begin{array}{cc} \left(\text{1}\;/m\right) & \sum_{i=1}^{m}{\bar{W}}^{i} \end{array}$$

### 3.3 Construct evaluation matrixes and perform fuzzy calculation

A fuzzy matrix $R=\left(rij\right)m\times n$, as is shown in formula (3), is obtained by fuzzy linear transformation, $rij=\frac{{\text{the number of the indicator number to select the level v}}_{i}}{\text{the number of participating evaluation}}$.

(3) $$R=\left(rij\right)m\times n\left[\begin{array}{cccc} r11 & r12 & \cdots & r1n\\ r21 & r22 & \cdots & r2n\\ \vdots & \vdots & \vdots & \vdots \\ rm1 & rm2 & \cdots & \mathrm{rmn} \end{array}\right]$$

Then, the overall evaluation vector is established. The overall evaluation vector $U_{i}$, as is shown in formula (4), can be obtained based on the first‐level evaluation matrix and fuzzy matrix.

(4) $$U_{i}=W_{i}\cdot R=\left(w_{i1},w_{i2},\cdot \cdot \cdot ,w_{\mathrm{im}}\right)\cdot \left[\begin{array}{cccc} r11 & r12 & \cdots & r1n\\ r21 & r22 & \cdots & r2n\\ \vdots & \vdots & \vdots & \vdots \\ rm1 & rm2 & \cdots & \mathrm{rmn} \end{array}\right]=\left(u_{1},u_{2},u_{3},u_{4},u_{5}\right)$$

Finally, the evaluation set that this paper selects is V = {good, relatively good, general, relatively poor, poor}, and the quantified value set that is *N* = {100, 75, 50, 25, 0}. The final performance evaluation index F, as is shown in formula (5), is obtained by weighted average.

(5) $$F=100\times u_{1}+75\times u_{2}+50\times u_{3}+25\times u_{4}+0\times u_{5}$$

## 4 THE SURVEY AND THE DATA

### 4.1 Questionnaire investigation

#### 4.1.1 Questionnaire design

According to the index system of FSSP mentioned in Table S1, the Government Food Safety Supervision Performance Questionnaire is designed. The five‐grade classification method is used to score each item in the questionnaire: “good” means 100 points, “relatively good” means 75 points, “general” means 50 points, “relatively poor” means 25 points, and “poor” means 0 point. Each item is assigned a corresponding level of five scoring criteria to ensure the objectivity of scoring. Further, the task group randomly selected Guangdong and Henan as the pilots for a preliminary research, and ultimately the questionnaire is determined.

#### 4.1.2 Sample

FDA is the official government department that is in charge of food and drug management, and supervises the implementation of various systems and standards under the subordinate local governments according to the laws and regulations. Additionally, as the official regulatory authority, FDA covers the central, provincial, prefectural, and county‐level administrative units (At the central level, it refers to CFDA, China Food and Drug Administration). Therefore, taking the sample from the FDA will ensure the scientific nature of the original data acquisition, which contributes to objective evaluation of China's FSSP.

The survey was conducted in June 2016 and lasted for four months. The research group was composed of the professors of food safety management from different colleges and universities, as well as the graduate students who have been trained in food safety management. The data were collected at the end of September 2016. To ensure the objectivity of the results, the data were obtained from the official websites of FDA or via telephone survey and the score was strictly based on the criteria. In this study, a questionnaire was on behalf of a food safety regulatory body and a total of 697 questionnaires were administered, among which seven were invalid and 690 were effective. The effectivity rate was 98.996%, and 20,010 valid survey data were obtained.

### 4.2 Sample characteristics

The survey involves 690 FDA of four administrative levels, and the distribution and characteristics of the sample are shown in Tables S2 and S3 refer to appendix. In addition, in Table S3, for the convenience of statistics and analysis, the central is compared in statistics. Consequently, the central and provincial results appear side by side. At the central level, research group only investigated China Food and Drug Administration (CFDA).

### 4.3 Test of reliability and validity

In this paper, SPSS19.0 statistical analysis software is used to analyze the reliability of the questionnaire, as shown in Table S4 refer to appendix. Cronbach's alpha values of presupervision, internal supervision and postsupervision are 0.961, 0.987, and 0.983, all of which are above 0.550 in general, indicating that the questionnaire has good internal consistency and stability, and the reliability is quite good. Meanwhile, the construction validity of questionnaire is tested by confirmatory factor analysis, and the KMO values of presupervision, internal supervision, and postsupervision are above 0.9, indicating that the relevance of factor analysis is quite good and the validity is quite high.

## 5 RESULTS AND DISCUSSION

### 5.1 Evaluation results

With the help of ANP structure, Delphi expert scoring and the Super decision software, the weight of the FSSP indexes is determined using Super Decision software (Table S5 refer to appendix). Further, according to the system analysis of the 690 questionnaires, this paper utilizes ANP‐fuzzy comprehensive evaluation model, and then obtains China's FSSP. The scores in different supervision links, administrative levels and provinces are shown in Tables S6–S8 refer to appendix.

## 6 DISCUSSION

As shown in Table S6, the overall score of FSSP in China is 60.350, and the score of presupervision, internal supervision, and postsupervision are respectively 61.125, 52.750, and 67.250. Table S6 shows that the overall situation of food safety is stable and controllable, which is consistent with the judgment made by Li Keqiang, Premier of State Council, on the current situation of food and drug safety in China. However, deficiencies of the government's supervision in presupervised food safety risk, food recall, food safety accident summary, and investigation afterward can be seen and affect the overall level of FSSP in China. Reviewing the “melamine” incident, regulatory authorities lacked the necessary risk monitoring and assessment system for food safety, and the implementation of the food recall system was not in place. Moreover, after the outbreak of the incident, the local authorities were even secretive, resulting in great reputation and economic losses in the food industry in China.

As shown in Tables S6–S8, from the different supervision links and administrative levels and provinces, the performance of the regulatory process is poorer than that of the prior prevention and transaction. In the practice of food safety supervision, the supervision department pays more attention to the perfection of relevant laws and regulations of food safety in advance as well as the subsequent responsibility. However, the implementation of laws and regulations and supervision system tends to be deviated, resulting in lower FSSP level. For example, in November 2011, the “bacterial gate” incident occurred in Sanquan Foods Co., Ltd, and due to the negligence of government regulators, the issue of the food problem has not been recalled. In conclusion, in the case of the lack of government supervision, the loss of supervision such as that in food recall in the food safety supervision system is particularly serious.

As shown in Table S7, CFDA’s FSSP obtains the highest score, which is 88.093, and the scores of the provincial and prefecture level administrative regions are 75.804 and 68.625, respectively, while the score of the county‐level administrative region is 48.590. Thus, with the decline in the administrative level, the performance level on government's food safety supervision as a whole and for each link that has been decreasing can be seen. The quality of the supervision team and investment is different because they are from different administrative levels, causing the grassroots government food safety supervision to become a weak area in China. This is consistent with the requirements that make up the weakness of food safety supervision in grassroots units in 2016 Food Focus.

Table S8 shows that, except for CFDA and other municipalities, Guangdong, Shaanxi, Anhui, and Yunnan obtain a high score, achieving a higher ranking. Heilongjiang, Xizang, and the other eight provinces obtain a poor score, obtaining a lower ranking. In addition, Table S8 shows that the FSSP level of Shaanxi, Qinghai, Gansu, and other western provinces exceeds that of the Shandong, Hubei, Hunan, Henan, and other central provinces. Shaanxi province, especially ranks sixth, which is far more than Jiangsu, Zhejiang, Fujian, and other economically developed provinces in East China. To sum up, there is no positive correlation between food safety control and regional economic developmental level, and the assumption does not match.

## 7 CONCLUSION

According to the constructed the index system of FSSP, we utilize the analytic network process‐fuzzy comprehensive evaluation model (ANP‐fuzzy) to conduct an empirical analysis of government supervision performance. This research shows that (a) the overall situation of China's food quality and safety is controllable, but the government does not do well in supervision of food safety risk, food recall, and accident summary. (b) Regulatory mechanisms are not in place, and the lack of regulation makes internal supervision the weakest link in FSSP. (c) Grassroots supervision is weak, and FSSP gradually declines with that decrease in the administrative level; (d) The developing level of economy and regulatory level in a region have no positive correlation. If local governments have low awareness and do not pay attention to food safety supervision, economically developed areas may break out in numerous food safety accidents.

Despite a great deal of work, there exist some inadequacies in the aspect of longitudinal dynamic comparative analysis, for the paper merely collected the FSSP data from FDA in 2016. Therefore, the future research will not only concentrate on the continuous investigation into the original target but also track the continuous changes of FDA’s food safety supervision performance, thus able to enhance the government's self‐supervision ability and protect the public's rights to know the food safety information.

## CONFLICT OF INTEREST

The authors declare that they have no competing interests.

## ETHICAL STATEMENT

This study does not involve any human or animal testing.

## Supporting information

Table S1

Table S2

Table S3

Table S4

Table S5

Table S6

Table S7

Table S8
